# Preventively enteral application of immunoglobulin enriched colostrums milk can modulate postoperative inflammatory response

**DOI:** 10.1186/2047-783X-18-50

**Published:** 2013-11-23

**Authors:** Klaus Orth, Wolfram Trudo Knoefel, Martijn van Griensven, Christiane Matuschek, Matthias Peiper, Holger Schrumpf, Peter Arne Gerber, Wilfried Budach, Edwin Bölke, Bettina Alexandra Buhren, Matthias Schauer

**Affiliations:** 1 Medical Faculty, Department of General, Visceral, and Thoracal Surgery, Asclepios Harz Hospitals, Goslar, Germany; 2 Medical Faculty, Department of General, Visceral-, and Pediatric Surgery, Heinrich Heine Universität Düsseldorf, Germany University of Düsseldorf, Dusseldorf, Germany; 3 Department of Trauma Surgery, Klinikum rechts der Isar, Technische Universität München, Munich, Germany; 4 Medical Faculty Department of Dermatology, Heinrich Heine Universität Düsseldorf, Germany University of Düsseldorf, Dusseldorf, Germany; 5 Medical Faculty Department of Radiation Oncology, Heinrich Heine Universität Düsseldorf, Germany University of Düsseldorf, Moorenstrasse 5, Duesseldorf D-40225, Germany; 6 Klinik für Allgemein-, Viszeral-, Gefäß- und Unfallchirurgie, Krankenhaus St. Joseph. Propsteistr. 2, Essen-Werden 45239, Germany

**Keywords:** Inflammatory response, Endotoxin translocation, Acute phase response

## Abstract

Several studies demonstrated acute inflammatory response following traumatic injury. Inflammatory response during surgical interventions was verified by a significant increase of endotoxin plasma levels and a decrease of the endotoxin neutralizing capacity (ENC). However, the incidence of elevated endotoxin levels was significantly higher (89%) than detected bacterial translocation (35%). Thus parts or products of Gram-negative bacteria seem to translocate more easily into the blood circulation than whole bacteria. Along with the bacterial translocation, the inflammatory response correlated directly with the severity of the surgical intervention. In comparison after major and minor surgery Interleukin-6 (IL-6) and C-reactive protein (CRP) was also significantly different. Similar effects in mediator release were shown during endovascular stent graft placement and open surgery in infrarenal aortic aneurysm. Open surgery demonstrated a significant stronger endotoxin translocation and a decrease of ENC. Strategies to prevent translocation seem to be sensible. Colostrum is the first milk produced by the mammary glands within the first days after birth. It contains a complex system of immune factors and has a long history of use in traditional medicine. Placebo-controlled studies verified that prophylactic oral application of immunoglobulin-enriched colostrum milk preparation diminishes perioperative endotoxemia, prevents reduction of ENC and reduces postoperative CRP-levels, suggesting a stabilization of the gut barrier. This effect may be caused by immunoglobulin transportation by the neonatal receptor FcRn of the mucosal epithelium.

In conclusion, there is an association of perioperative endotoxemia and the subsequent increase in mediators of the acute phase reaction in surgical patients. A prophylactic oral application of colostrum milk is likely to stabilize the gut barrier i.e. reduces the influx of lipopolysaccharides arising from Gram-negative bacterial pathogens and inhibits enterogenic endotoxemia. This appears to be a major mechanism underlying the therapeutic effect in patients at risk for Gram-negative septic shock.

## Review

Multiple studies have demonstrated endotoxin as the most crucial pathogenic factor of Gram-negative bacteria and its role in Gram-negative sepsis [1-20]. Endotoxemia was shown to occur often following traumatic injury and shock, and in a variety of chronic diseases. Notably, surgical interventions are also known to be associated with an increased release of inflammatory mediators, depressed immune function and increased susceptibility to subsequent infection (Figure 1). Various studies have shown a correlation between the extent of the surgical intervention and the inflammatory response [4,21-24]. Herein, the postoperative acute-phase reaction is induced by the translocation of bacterial products in the gut causing an inflammatory response with a stress reaction and secretion of catecholamines [18,25]. Likely, endotoxin translocation plays a major role in triggering infectious complications in trauma and surgical patients [26,27]. Preventive protection of the mucosal barrier functions by selective decontamination with antibiotics and nutritional strategies have proven to be beneficial [4,22,28-32]. Furthermore, the enteral applications of an immunoglobulin-enriched colostrum preparation stabilize the gut barrier and diminish the peri- and postoperative endotoxin translocation and consecutively, the acute phase response (Figure 1) [22,33] (Table 1).

**Figure 1:** **Interaction of endotoxin translocation and acute phase response.** Diminished acute phase response in patients with less endotoxin translocation by immunoglobulin impact.

**Table 1:** Summary of the crucial literature

[4]	Boelke E *et al*.; Wien Klin Wochenschr 2002	Immunoglobulin-enriched colostrum milk preparation reduces endotoxin translocation and acute phase response in cardiac patients.
[7]	Hsiao HB; Shock 2011	Kinsenoside suppresses LPS-stimulated inflammatory reactions
[22]	Bolke E; Angiology 2001	Changes of gut barrier function during cardiac surgery
[34]	Struff WG; Int J Clin Pharmacol Ther 2007	Inhibition of intestinal LPS absorption measured after bovine colostrum milk application diminises IL-6 and CRP
[35]	Deitch EA; Front Biosci 2006	The gut-lymph hypothesis, reduction of endotoxin binding protein in surgery patients
[36]	Brandtzaeg P; Springer: New York, NY, USA 2007	IgA agglutination of microbes, adherence and invasion of mucosal epithelial cells
[37]	Fernandez MI; Immunity 2003	Internalization of IgA into intestinal epithelial cells
[38]	Olah A; Hepatogastroenterology 2007	Enteral nutrition reduces sepsis in patients with pancreatitis
[39]	Friedrich I; Eur J Med Res 2002	IgM-enriched immunoglobulin preparation for immunoprophylaxis in cardiac surgery
[40]	Fujitani K; Br J Surg. 2012	Prospective randomized trial of preoperative enteral immunonutrition followed by elective total gastrectomy for gastric cancer

LPS, lipopolysaccharide; CRP, C-reactive protein; IgA and IgM, immunoglobulin A and M.

Colostrum has a long history of medicinal use. It is the first milk produced by the mammary glands within the first days after birth. Bovine colostrum is homologous to human colostrum, although the protein content is about twenty-, and the amount of immunoglobulin (Ig)G about ten-times higher than that of the human equivalence [41,42]. Bovine colostrum is accepted for human use and can easily be produced in large quantities [41]. It contains large amounts of immunological factors to support growth and immune maturation of the digestive tract and provides passive immunity until the newborn has synthesized its own active immune defense system [41,43-48]. Beside nutrients such as carbohydrates, amino acids, fat, vitamins, and minerals colostrum contains Ig, including IgG, IgM and IgA, which may provide a defense in both the treatment and prevention of viral and bacterial infections [34,49,50]. Bovine IgG from colostrum or milk can be effective as a means of providing passive immunity to protect animals and humans from diseases. The immunoglobulins found in milk and the transfers of passive immunity from mother to neonate (Figure 2) have been reviewed by a number of authors, with a partial listing of references [50-68].

**Figure 2:** Immunoglobulin resorption by the neonatal Fc receptor (FcRn) in mucosal epithelia.

The inflammatory response with its adverse aspects still remains an only partially understood, unresolved problem after large surgical interventions. However, the use of monoclonal and polyclonal antibodies in therapy in humans has made them the fastest-growing protein pharmaceutical agent. Our objective was to re-evaluate postoperative endotoxemia, its impact on postoperative inflammatory response and the interaction of colostrum milk immunoglobulin on the postoperative course as a possible treatment.

### Inflammatory response during abdominal, general and vascular surgery

Boelke *et al*. [21] measured plasma endotoxin levels, endotoxin neutralizing capacity (ENC) and plasma levels of endotoxin-binding proteins (transferrin, alpha-2-macroglobulin, albumin, apo-A, apo-B, IgG, IgA and IgM) in 25 patients with thyreoidectomy and 52 patients with abdominal surgery during and after surgery, in order to evaluate the association of endotoxemia and inflammatory response in correlation with minor and major surgical interventions.

Strikingly, plasma levels of endotoxin showed an increase in the early phase of elective surgical interventions, most likely due to loss of the intestinal barrier function. In the major surgery group plasma levels of endotoxin increased immediately after application of anesthesia, whereas in the minor surgical group, endotoxin plasma levels increased after skin incision. The early increase in the major surgical group may be due to more severe anesthesiological manipulation. The relative increase in endotoxin plasma levels was significantly higher (area under the curve (AUC), *P* <0.005) in the major surgery group as compared to the group subjected to minor surgery. The ENC, a parameter for the ability to clear systemic endotoxin, decreased significantly during surgery in both groups, and to a significantly larger extent in patients receiving major surgery (AUC, *P* <0.05).

Deitch *et al*. [35,69-73] identified the gastrointestinal tract as the major source of plasma endotoxin. However, there was no significant difference between colonic surgery and other abdominal interventions in the major surgery group related to endotoxin plasma levels or endotoxin-binding proteins (EnBP). Also, bacterial translocation was similar in both groups [e,f,g]. Thus direct contamination of the peritoneal cavity during colonic surgery did not play an important role. Bacterial translocation to mesenterial lymph nodes in the major surgery group occurred in 35%, whereas endotoxin plasma levels were elevated in 89% of patients in this group [21]. In conclusion, parts or products of Gram-negative bacteria seem to translocate more easily through the gut mucosa than whole bacteria.

Several studies have shown that the perioperative increased plasma endotoxin level activates the release of inflammatory mediators [70,74,75]. IL-6 increased with a distinct delay after the observed changes of endotoxin plasma levels with a significantly higher plasma level in the major surgical group (Figure 1). Similarly, another study could show that the severity of the traumatic impact or surgical intervention correlates with the subsequent increase in IL-6 levels, inducing a major increase of C-reactive protein (CRP) [21,23].

Similar results were found in 42 patients in whom endotoxin release was compared during open, versus laparoscopic, gall bladder surgery. The laparoscopic group had higher ENC, lower plasma endotoxin, and consequently a stronger postoperative acute-phase reaction with higher CRP levels. Therefore, the extent of the surgical approach with the same extent of surgical resection, without bowl resection or manipulation, correlated positively with endotoxemia and subsequently with the intensity of the acute-phase reaction.

The same results were found in aortic surgery. Mediator release (IL-6, CRP) during endovascular stent grafts of infrarenal aortic aneurysms was significantly lower when compared to that during open surgery [23]. From the beginning of the open surgical procedure, endotoxin and ENC levels increased and peaked at the end of the operation. However, patients with endovascular stent grafts had a significantly lower delayed increase of plasma endotoxin and ENC levels. Similar to the comparison of open versus laparoscopical cholecystectomy, the difference in endotoxemia depended on the surgical approach followed by a subsequent significantly lower production of acute-phase mediators in the non-intestinal surgical intervention.

In contrast to other authors Moore *et al*. did not find bacterial translocation after severe injury and hemorrhagic shock [76-78]. They inserted portal vein catheters for sequential blood sampling in the operating room, at 6, 12, 24, and 48 hours, and 5 days postoperatively in 20 injured patients requiring emergency laparotomy. Twelve patients (60%) arrived at the hospital in shock (SBP <90 torr). Eight of 212 (2%) portal blood cultures were positive, seven cultures were presumed contaminants. Within the first 48 hours, they could not detect endotoxin in portal or systemic blood. Simultaneously obtained portal and systemic blood levels of complement fragment C3a, TNF, and IL-6 were nearly identical and not different in those patients who developed multiple organ failure. In this prospective clinical trial neither portal nor systemic bacteremia were confirmed within the first 5 days post injury, despite major torso-trauma and a high incidence of shock.

Although bacterial translocation has been consistently demonstrated in many studies and experimental models, its occurrence or detection in humans seems to be uncertain [76-82]. Secondary endotoxemia appears to be the most plausible link. However, its precise role and specific mechanisms of initiating distant organ dysfunction remain to be acknowledged. Probably the same elements that favor bacterial translocation promote escape of their toxic cell membrane from the gut lumen. With regard to these considerations, strategies have been developed to prevent endotoxin translocation by stabilizing the barrier dysfunction, that is, by selective bowel decontamination with antibiotics and oral application of Ig.

### Interactions of colostrum and milk immunoglobulins in the intestine

Immune milk products have protective effects on neonatal, infant, and adult human health. The exact function and the effects of immune milk products are less clear and require further investigations. Colostrum and milk contain Ig, and a range of antimicrobial products and factors that may impact on the immune system [1,41,83-90]. These factors include leukocytes, macrophages and lymphocytes. In addition, colostrum and milk contain antibacterial enzyme lactoperoxidase, antibacterial and lytic enzyme lysozyme, oligosaccharides that function as equivalents of microbial ligands on mucosal surfaces, antimicrobial heat-stable peptides and soluble CD14, and the iron-binding antimicrobial protein, lactoferrin. Colostrum contains cytokines and growth factors, which may affect the neonatal intestinal development and intestinal immune responses to disease in adults [90,91]. This provides a source of energy that may impact IgG absorption in the neonate [92]. All these factors vary considerably among different species. Maternal antibodies may inhibit infant responses to vaccine administration and effect the development of the infant’s immunity [93].

Most macromolecules are degraded by digestive enzymes, but a portion of macromolecule is transported through the intact intestinal wall, including protein [94,95]. It is therefore expected that a large part of consumed Ig is either partially or completely digested. However, a portion of the Ig remains intact and capable of binding to an antigen (Figure 2) [68].

Secretory IgA (sIgA), which is present in milk and colostrum, is the primary Ig for immune protection of the mucosal membranes, such as the intestine. This may contribute to the protective effects of these secretions [36], which have antimicrobial properties such as agglutination of microbes and neutralization of viruses. Furthermore, a non-inflammatory extracellular and intracellular immune defense by inhibition of adherence and invasion of mucosal epithelial cells has been observed [36,68]. Secretory IgA neutralizes pathogens in the intestinal lumen [96]. Bacterial enterotoxins can be neutralized by binding and internalization of sIgA into intestinal epithelial cells [37]. Intracellular immunity is based on transcytosed sIgA by the enterocytes, neutralizing viral particles within the endosomic system (Figure 2) [7].

IgA has a major role in the immunosuppressive mechanisms in the intestine wall that inhibit proinflammatory responses to oral antigens [36]. This suppression is compensated by systemic immune factors, including systemic IgG, which results in inflammation and tissue damage once an antigen crosses the epithelial barrier to the lamina propria [36]. Any IgG localized in the lamina propria, whether from systemic sources or from the intestinal lumen, initates proinflammatory responses in the intestine wall [36]. In this context, balancing IgG-antigen immune complexes to the lamina propria for immune processing were investigated [36,97].

Further on, the intestinal mucus layer does provide an important protective barrier in the interactions of the intestinal tissue with microbes [98]. Functionally intact IgG that remains in the intestinal lumen is expected to bind antigens and participate in protection of the tissue through immune exclusion. In this context, an IgG Fc binding site has been identified in association with the intestinal mucus [99-101]. The Fc binding protein can block the passage of IgG-antigen complexes to the enterocyte surface, thereby blocking its uptake and transport to the lamina propria. In this way the complexes are degraded in the intestinal lumen followed by excretion [91,101].

The usual daily dose of the commercially available bovine colostrums preparation, Lactobin® is 10 to 20 g daily. Higher doses can be used in the majority of patients because of low incidence of intolerance problems. Clinical trials have provided evidence that oral application reduces the input of lipopolysaccharides (LPS) from the gut [21]. This appears to be a major mechanism underlying its therapeutic effect in patients at risk for Gram-negative septic shock.

### Preoperative oral application of immunoglobulin-enriched colostrum milk in patients with abdominal surgery

Based on findings of the postoperatively induced acute-phase reaction by bacterial product translocation, strategies to prevent endotoxin translocation, that is, by oral application of Ig were developed. It is well-known that enteral application of IgA-enriched milk reduces the incidence of necrotizing enterocolitis in premature babies by stabilizing the barrier dysfunction of the immature gut [74]. In consideration of this reduction, enteral application of an Ig-enriched colostral preparation was evaluated to diminish the peri- and postoperative endotoxin translocation in patients undergoing abdominal surgery.

The impact of immunoglobulin feeding on mediator responses was analyzed in 40 patients undergoing major abdominal surgery [22]. The placebo-controlled determination of endotoxin and ENC was performed using a chromogenic modification of the limulus amebocyte test. IL-6 levels were determined by ELISA. CRP and endotoxin-binding proteins (transferrin, alpha-2-macroglobulin, albumin apo-lipoprotein A1, B, IgG, IgA and IgM) were measured nephelometrically. With abdominal surgery, the study revealed a significant reduction of circulating endotoxin levels through gut stabilization by enteral application of IgA-enriched milk with decreased inhibition of plasma ENC. The maximal loss of ENC was reduced and recovery was accelerated by colostral milk. Comparing the AUC in both groups, a highly significant improvement of ENC was found in gut barrier-stabilized patients (*P* <0.05) [22]. As ENC indicates cumulative effects, the indirect determination of endotoxemia by assessing the ENC of plasma was more sensitive than the determination of endotoxin by a limulus amebocyte test.

Endotoxemia represents a trigger of acute-phase reaction proteins such as IL-6 and CRP [22]. IL-6 has been shown to peak 6 hours after surgery, and CRP to peak on the second day. Lower serum levels of both proteins were measured in the colostrum group (Figure 1). Due to the wide variance, serum levels did not reach statistical significance. Similar observations were made after selective bowl decontamination. However, in the case of incomplete decontamination, a minor degree of reduction in peri- and postoperative endotoxemia was found, which did not fully explain the reduction of IL-6 plasma levels. Therefore, preoperative oral application of Ig-enriched colostral milk in patients with major abdominal surgery significantly reduces the amount and the duration of endotoxemia and ENC. This effect is likely due to a stabilization of the gut barrier.

These results are in accordance with those of other studies undergoing gastric and pancreatic surgery with live or heat-inactivated lactic acid bacteria [102]. The authors noted a one-month sepsis rate with live *Lactobacillus plantarum 299* (*L. plantarum*) in one of fifteen, compared with three of seventeen patients who received heat-inactivated *L. plantarum*. Of 16 patients who received parenteral nutrition with fermentable fiber and no lactobacillus, 8 developed sepsis (*P* = 0.001). A large controlled study of patients with pancreatitis showed that enteral nutrition significantly reduced septic complications, but made no difference to the rate of multiple organ failure or death [38,103]. Similar results were obtained in patients undergoing liver transplantation, showing a significant reduction in sepsis rates and an improved surgical outcome [104]. Of 31 patients who received live *L. plantarum 299* and fermentable fiber, 4 developed infections, compared with 11 of 34 who were given heat-killed *L. plantarum 299* and fiber, and 15 of 32 were treated with selective bowel decontamination (*P* = 0.017). Well-controlled clinical studies in a total of 100 surgical patients showed that the inhibition of intestinal LPS absorption measured after bovine colostrums-concentrate applications not only reduced LPS levels in the peripheral blood, but also diminished inflammatory parameters such as IL-6 and CRP [34].

### Preoperative oral application of immunoglobulin-enriched colostrum milk in patients with cardiac surgery

Patients were found to have elevated endotoxin plasma levels during abdominal surgery. Endotoxemia occurs commonly and can be one reason why patients develop infectious complications after surgery [21,105]. In patients who underwent cardiac surgery, endotoxin plasma levels correlated with the catecholamine required to obtain the necessary hemodynamic conditions during surgery [22]. Previous studies in cardiac patients demonstrated that the severity of endotoxemia is reduced by perioperative selective decontamination of the gastrointestinal tract, indicating that endotoxin translocation from the gastrointestinal tract is essentially involved [22,106].

In a prospective placebo-controlled study, 30 out of the 60 patients who had cardiac surgery received immunoglobulin-enriched colostrum milk two days preoperatively. Endotoxin and ENC levels were elevated at the end of the operation. This seemed to have had a trigger function for the acute-phase response [4]. However, no reductions of endotoxin plasma levels, ENC or IL-6 levels were observed in the colostrum milk group throughout the observation period. CRP-levels in all patients peaked 48 hours after the operation but was lower in the verum group (*P* = 0.034). Similar to the abdominal surgery study, endotoxemia was detected at an early stage within an elective cardiac operation. Endotoxemia was followed by a subsequent increase in mediators of the acute-phase reaction. The prophylactic enteral application of a bovine milk preparation for two days in cardiac patients reduced postoperative plasma CRP levels, but did not reduce perioperative endotoxin, which does not support the abdominal surgery observations. The different perfusion of the bowel during cardiac surgery or the small amount of colostrum preparation administered could present one explanation. On the other hand, not all antibodies directed against pathogenic bacteria (anti-LPS) are available in Lactobin®. This can lead to partial reabsorption of specific LPS molecules from the intestine despite Lactobin® treatment [4].

Friedrich *et al*. [39] randomized 41 cardiac surgical patients into two groups receiving either an IgM-enriched preparation combined with routine antibiotic prophylaxis or routine antibiotic prophylaxis plus placebo. Patients were comparable with respect to their Acute Physiology and Chronic Health Evaluation (APACHE) II score, coronary risk, comorbidity, operating time, clamping time, and ischemic time. Even though no significant endotoxin plasma levels were detected in either group, ENC levels reached significance. However, IL-6, TNF-alpha, IL-10 and TNF-R1 were not different in both groups. There were significantly fewer patients with signs of inflammation (fever, leukocytosis, hypotension) in the treated group (*P* <0.05), which was further related to a reduced hospitalization period (12.1 versus 13.0 days).

Another study by Fujitani *et al*. [40] randomized 244 patients with gastrectomy for gastric cancer into two groups: 127 patients preoperatively received immunonutrition, and 117 patients were randomized into a control group. The postoperative clinical course, infectious complications, sepsis and postoperative inflammatory mediators (for example, CRP) did not show a significant difference when comparing both groups. As the results are very different in many studies [107], the type of immunonutrition seems to play an important role. Currently, routine use of immunonutrition cannot be recommended because of insufficient evidence.

## Conclusion

Enteral nutrition is not just the acquisition of calories and nitrogen, but it also offers the possibility of the acute-phase response modulation and immune-function improvement. Benmark [108] noted 75% immune-function localization in the gastrointestinal tract. This offers nutritional science a window to modulate this system. A bacterial translocation could not always be proven in patients after major trauma. Moore *et al*. did find significant bacteremia or endotoxemia in their study of 20 patients [76]. However, several investigations demonstrated the impact of perioperative endotoxemia and subsequent activation of acute-phase mediators, such as IL-6 and CRP, in patients with intestinal, general, vascular and heart surgery. Bacterial translocation and endotoxemia does not only occur in patients after colonic surgery but also in all other surgical interventions. Therefore, the impact is associated with the extent of the surgical intervention and the surgical approach (open surgery versus minimal invasive treatment). Preventive protection of the mucosal barrier function by selective decontamination with antibiotics was proven to be beneficial. However, selection and mutation of bacteria interdict a non-selective application of antibiotics. Therefore, nutritional strategies are favorable as they were proven to be effective and they do not promote selective breeding of resistant bacteria. The main actions include an antibacterial effect and the modulation of the immune response. Polyvalent bovine colostrum concentrates are able to neutralize LPS, that is, endotoxins arising from Gram-negative bacterial pathogen, and can inhibit activation of acute-phase mediators.

The concentration in colostrum of specific antibodies against pathogens is raised by immunizing cows with these pathogens or their antigens. Immune milk products are supplements made of such hyperimmune colostrum or antibodies enriched from this milk. These products can be used to give effective specific protection against different enteric diseases and are commercially available for animal farming. They were also proven to be effective in balancing gastrointestinal microbial flora and in prophylaxis against various infectious diseases in humans. Positive results have been obtained with products targeting *Rotavirus*, *Shigella flexneri*, *Escherichia coli*, *Clostridium difficile*, *Streptococcus mutans*, *Cryptosporidium parvum* and *Helicobacter pylori*. Clinical studies are currently in progress to evaluate the efficacy of immune milks in the prevention and treatment of various human infections, including those caused by antibiotic-resistant bacteria. Immune milk products are promising examples of health-promoting functional foods.

## Abbreviations

AUC: Area under the curve; CRP: C-reactive protein; ELISA: Enzyme-linked immunosorbent assay; EnBP: Endotoxin-binding protein; ENC: Endotoxin neutralizing capacity; IL: Interleukin; Ig: Immunoglobulin; sIgA: Secretory immunoglobulin A; TNF: Tumor necrosis factor.

## Competing interests

All authors disclose any potential financial, professional, or personal conflict that are relevant to this manuscript. We disclose funding received for this work from the National Institutes of Health (NIH), Wellcome Trust, and others.

## Authors’ contributions

All authors were involved in drafting or revision of the manuscript and intellectual input. All authors read and approved the final manuscript.
